# Potential of Black Phosphorus in Immune-Based Therapeutic Strategies

**DOI:** 10.1155/2022/3790097

**Published:** 2022-07-11

**Authors:** Wenjuan Dong, Hu Wang, Hailin Liu, Chunqiao Zhou, Xuelin Zhang, Song Wang, Lin He

**Affiliations:** ^1^Department of Pharmacy, The First People's Hospital of Chongqing Liang Jiang New Area, Chongqing 401121, China; ^2^Department of Pharmacy, Sichuan Academy of Medical Sciences & Sichuan Provincial People's Hospital, School of Medicine, University of Electronic Science and Technology of China, Chengdu 610072, China

## Abstract

Black phosphorus (BP) consists of phosphorus atoms, an essential element of bone and nucleic acid, which covalently bonds to three adjacent phosphorus atoms to form a puckered bilayer structure. With its anisotropy, band gap, biodegradability, and biocompatibility properties, BP is considered promising for cancer therapy. For example, BP under irradiation can convert near-infrared (NIR) light into heat and reactive oxygen species (ROS) to damage cancer cells, called photothermal therapy (PTT) and photodynamic therapy (PDT). Compared with PTT and PDT, the novel techniques of sonodynamic therapy (SDT) and photoacoustic therapy (PAT) exhibit amplified ROS generation and precise photoacoustic-shockwaves to enhance anticancer effect when BP receives ultrasound or NIR irradiation. Based on the prospective phototherapy, BP with irradiation can cause a “double-kill” to tumor cells, involving tumor-structure damage induced by heat, ROS, and shockwaves and a subsequent anticancer immune response induced by in situ vaccines construction in tumor site, which is referred to as photoimmunotherapy (PIT). In conclusion, BP shows promise in natural antitumor biological activity, biological imaging, drug delivery, PTT/PDT/SDT/PAT/PIT, nanovaccines, nanoadjuvants, and combination immunotherapy regimens.

## 1. Introduction

Immunotherapy, which topped the list of 10 scientific breakthroughs in 2013 [1], is considered the fourth most common mainstream treatment mode of cancer following surgery, chemotherapy, and radiotherapy. Recently, a variety of immunotherapy strategies have been developed, including immune checkpoint inhibitors, adoptive-cell therapy, vaccines, adjuvants, targeted antibodies, cytokines, and oncolytic viruses [2, 3]. In addition, a series of advances have recently been made in cancer immunotherapy. For example, Li et al. discovered that gut microbes can enhance the antimelanoma effect of immune checkpoint inhibitors [4]. However, although immunotherapy has brought revolutionary advances in cancer treatment, not all patients can derive clinical benefits from it [5, 6]. For example, pembrolizumab, a PD-1 inhibitor, is only effective for approximately one-third of patients with nonsmall cell lung cancer [7]. With the understanding of immunotherapy and immunosuppression, researchers identified several mechanisms involved in immune escape and drug resistance, such as downregulation of tumor antigen expression [8], upregulation of immune checkpoints in tumor cells or exosomes [8], insensitivity to immune effector molecules [8], tumor-associated immunosuppressive factors [8], cells in the tumor microenvironment (TME) (the abbreviation) [9], and angiogenesis in tumor [10] or gut microflora [4, 11]. To overcome these challenges, the need to find novel therapeutics is urgent.

In recent years, nanomedicine, a technology that employs materials ranging in size from 10 to 200 nm for imaging, diagnosis, and treatment of diseases [12], has shown great potential and promise in the field of cancer immunotherapy. As delivery systems, nano-biomaterials are ideal platforms for loading tumor antigens, vaccines, and adjuvants as well as immune checkpoint agents. In 2019, Wen et al. summarized numerous developed biodegradable nanocarriers, including polymer materials, lipid materials, biomacromolecules, and hybrid materials [13], which play important roles in promoting immune responses. Researchers also found that some nanomaterials have immunoadjuvant activity, such as graphene oxide modified with Au (GO-Au) [14]. Not only that, the surface modification potential of nanoparticles is also critical to boost an antitumor immune response. Rosalia et al. demonstrated that CD40-decorated nanoparticles coencapsulating Ag and Pam3CSK4 significantly enhance T cell immune responses [15]. The immune activity of nano-biomaterials has also been explored by researchers in recent years. For example, Jiang et al. discovered that NaCl nanoparticles promote an antitumor immune response by inducing immunogenic cell death (ICD) [16]. In addition to the above applications, nano-biomaterials combined with other therapeutics, such as photothermal therapy and radiation, also show great potential for cancer immunotherapy [17–19].

One hundred years after it was first synthesized, in 2014, black phosphorus (BP) began to be noticed by scientists for its application after enthusiasm arose about research on other two-dimensional (2D) materials, such as graphene and transition metal dichalcogenides, as well as monolayer hexagonal boron nitrile [20]. The structure of BP is generally divided into layers of bulk and 2D material, both of which are composed of only phosphorus atoms [21]. The 2D BP monolayer consists of two atomic layers that form a honeycomb structure with zigzag and armchair conformations [22]. Unlike graphene, 2D BP possesses a band gap measuring 0.3 eV in its bulk and 2.0 eV in its monolayer structure [23]. Therefore, among the innovative generation of 2D nanomaterials, BP has more exploration potential than other 2D nanomaterials based on its semiconductor properties, optical properties, biological properties, mechanical properties, topological features, and thermo electrical properties [20]. In other words, 2D BP has favorable biocompatibility and biodegradability [24]. 2D BP has recently shown great potential as a nano-biomaterial in the biomedical field for applications including imaging [25], drug delivery [26], photodynamic and photothermal therapies, chemotherapy [27], and immunotherapy [28]. With the rise of cancer immunotherapy treatments, researchers have recently turned to 2D BP for immunotherapy purposes, such as innate immune activity, vaccine delivery, adjuvant properties, and photoimmunotherapy (PIT). The specific application of BP for an anticancer immune response will be reviewed in this paper, as shown in Figure 1.

## 2. The Structure and Biological Properties of BP

Bulk BP possesses a layered crystal structure, which is bonded through van der Waals forces. Single- or few-layer BP, also called 2D BP or black phosphorene [29], is obtained by exfoliating bulk materials or through chemical synthesis. Mechanical exfoliation, liquid exfoliation, chemical exfoliation, and chemical vapor transport growth can be applied to prepare 2D BP [20]. In a monolayer, phosphorus atoms covalently bond to three adjacent phosphorus atoms to form a puckered bilayer structure that contributes to its unique in-plane anisotropy, as shown in Figure 2(a) [30]. In the lateral view shown in Figure 2(b), the phosphorus atoms in same layer are connected through a short bond length of 0.2224 nm, while phosphorus atoms at the top are connected to the bottom through a long bond length of 0.2244 nm. In the top view, as shown in Figure 2(c), a zigzag is formed in the *y* direction, and armchair conformations are formed in the *x* direction [20]. Unlike graphene, BP possesses a layer-dependent band gap ranging from 0.3 eV in its bulk to 2.0 eV in its monolayer structure, which indicates excellent light absorption capacity [23]. The unique structure of anisotropy and band gap determines a wide range of properties, including electronic conductivity, optical properties, thermal properties, topological features, and mechanical behaviors [31, 32], which promote the application of BP in physical biomedical fields.

Phosphorus, an essential element in bone and nucleic acids [20, 33, 34], lays the foundation for the application of BP in biomedicine. BP is biodegradable and biocompatible, as it converts into nontoxic phosphates under physiological conditions [34]. Zhou et al. discovered that BP could effectively inhibit tumor cell proliferation by producing a large number of phosphate anions in tumor cells, while maintaining high biocompatibility in normal cells [35]. Therefore, with its biocompatibility, biodegradability, low-toxicity, band gap, and anisotropy, as well as a high surface to volume ratio, BP as biomaterial has shown a broad application prospect in cancer therapy in recent years. To date, nanostructures of BP applied in biomedical research mainly involve BP nanosheets and BP quantum dots (BPQDs) as well as BP nanoparticles [36]. However, BP is unstable when exposed to oxygen, light, and water, which restricts the preparation and application of BP. The degradation mechanism is divided into three steps [37]: (i) photo-generated electrons from the conduction band of BP are transferred into O_2_ to obtain O_2_^−^ under the excitation of light, and because the valence band maximum and conduction band minimum of monolayer BP are −5.46 and −3.95 eV, respectively, and the redox potential of O_2_/O_2_^−^ is −4.11 eV; (ii) O_2_^−^ overcomes the reaction barrier to form suspended O on the surface of BP and to form *P*=*O*; (iii) to form H-bonds between water molecules and O, P atoms are removed, which leads to the breakage of P-P.

## 3. The Functionalization of BP

Numerous strategies have been explored to improve the stability of BP based on its degradation mechanism as shown Figure 3. One strategy, called encapsulation, oxidizes the surface layer of BP to form P-O-P bonds, which are very stable [38]. In addition, chemical modification and element doping are also used to stabilize the structure of BP, as shown in Figure 4 and Table 1. Specific passivation measures are described in detail in the following section.

### 3.1. Encapsulation

Following the discovery of AlOx-encapsulated BP, numerous strategies to protect the surface of BP from degradation under ambient conditions have been studied, including employing 2D heterostructures, polymers, nanoparticles, and biomembranes to encapsulate BP nanosheets, BPQDs, BP transistors, and BP photodetectors. Currently, polymers, such as polymer (polymethyl methacrylate) (PMMA) [39], poly (2-hydroxyethyl methacrylate)-co-poly (styrene) (PHMA-co-PS) [40], poly (1-hexyl-3-vinylimidazolium) hexafluorophosphate salt (PIL-TFSI) [41], and poly (ethylene glycol) (PEG) [42, 43], among others, exhibit the desired advantages to improving the stability of BP through encapsulation. For instance, PEG-encapsulated BP nanosheets showed not only excellent stability and dispersity, but also powerful application value in biomedical applications such as treatments for cancer and Alzheimer's disease [43, 44]. Additionally, Lu et al. constructed waterborne polyurethane (WPU) nanoparticles to encapsulate BPQDs to improve stability and dispersity, which contributed to BP-based photodynamic and photothermal therapy [45]. In recent years, biomembrane-coated nanoparticles, such as red blood cell membranes, cancer cell membranes, platelet membranes, exosomal membranes, and leukocyte membranes, give hope for the successful diagnosis and treatment of tumors [46]. It was also discovered that the encapsulation of BP into red blood cell membranes and cancer cell membranes, as well as exosomal membranes, not only promoted the blood circulation of BP, but also endowed BP with a targeting ability [47–49]. In addition, scientists also employ other 2D heterostructures, such as hexagonal boron nitride (hBN), graphene, and MoS_2_, to Sandwich BP [50].

### 3.2. Chemical Modification

The covalent chemical modification of BP is mainly led through nucleophilic substitution, radical reaction, or metal coordination to form P-X or P-O-X bonds [51]. For nucleophilic substitution, either BP reacts directly with alkyl halogens to form P-X, or chlorinated BP undergoes a reaction with thionyl chloride and then reacts with alkyl alcohol to form P-O-X [52]. Radical reaction is represented by aryl diazonium chemistry, such as 4-nitrobenzenediazonium salts (4-NBD) and 4-methoxybenzenediazonium tetrafluoroborate salts (4-MBD). Furthermore, modified diazonium, poly[(1,4-diethynylbenzene)-alt-9,9-bis (4-diphenylaminophenyl) fluorene] (PDDF), Nile Blue dye, and aryl iodonium salts are employed to enhance the stability of BP with desired dispersibility, additional dye function, and a higher degree of functionalization, respectively [53]. Sun et al. verified that P-C was successfully formed in covalent hybridization compounds as BP-graphite by free-radical reactions [54]. Although the formation of P-C or P-O-C bonds through diazonium functionalization or nucleophilic substitution can improve the stability of BP, there is still one unpaired electron in the phosphorus atom that inevitably restricts the passivation effect. Therefore, researchers creatively constructed *P*=*N* bonds by nitrene addition to BP with azide and achieved a passivation effect that was improved by about 4.7 times when compared with radical reaction BP with 4-NBD [55]. The covalent chemical modification of BP is different. For example, Zhao and colleagues reported that a titanium sulfonate ligand (TiL4) coordinated BP (TiL4@BPs) can significantly reduce the toxicity of BP and improve the stability of BP. In this metal coordination, the empty orbitals of titanium atoms in TiL4 were occupied by the lone pairs of electrons on BP to form coordination bonds [56].

Noncovalent modification has also been widely reported as another method for improving the stability of BP. At present, noncovalent chemical modifications of BP mainly involve three interactions: van der Waals interactions, cation-*π* interactions, and electrostatic interactions [53]. According to reports, 7,7,8,8-tetracyano-p-quinodimethane (TCNQ) and perylene diimides (PDI), as well as anthraquinone, are the commonly reported reagents to covalently modify BP through der Waals interactions [57–59]. Cation-*π* interactions are represented by noncovalently modified BP with silver ions (Ag^+^). Guo et al. demonstrated that passivated BP by Ag^+^ was stable in air, which provides the possibility of noncovalent modification of BP by other metal ions [60]. In addition to physical passivation methods, PILs-based protection strategies can also modify BP by electrostatic interactions, which enhance the stability of BP under ambient conditions for at least 100 days and maintain perfect stable performance of BP-based photodetectors for 120 hours [61].

### 3.3. Element Doping

In 2016, Yang et al. first reported that doping elements could improve the stability of BP [62]. They found that the incorporation of Te atoms reduces the conduction band minimum (CBM) of BP to make it difficult to form O_2_/O_2_^−^, which greatly slows down the degradation of BP in the environment. However, there are still some problems such as low yield and low doping concentration. Liu et al. discovered that short-distance transport growth strategy can transform red phosphorus into BP with a high conversion rate and high doping concentration. Various elements, such as As, Se, Te, Sb, Bi, Co, Fe, and Mn, can be doped into BP to promote air stability. Moreover, utilizing a transition metal, Sc doping also can bind to three P atoms on BP to form BP-Sc. Although the BP-Sc-2O structure is formed when BP is exposed to air, the redox potential of O2/O2^−^ (-4.11 eV) still exceeds the CBM of BP-Sc-2O (-4.75 eV), which contributes to its stability [63]. In addition to metal elements, Lv et al. also reported that the CBM of nonmetallic element S-doped BP was below the redox potential of O_2_/O_2_^−^, which prevented the oxidative degradation of BP in ambient conditions [64]. Compared with single element doping, Li et al. found that doping with two or three elements showed a better effect on promoting the stability of BP [65]. Therefore, it is possible to improve the stability of BP in ambient conditions and further promote the application of BP in physical biochemistry using these modified strategies.

## 4. BP-Based Therapeutic Strategies

### 4.1. BP-Based Photodynamic Therapy and Photothermal Therapy

In recent years, photothermal therapy (PTT) and photodynamic therapy (PDT), which can convert near-infrared (NIR) light into heat-energy or reactive oxygen species (ROS) to cause structural damage of tumor cells, have gradually become an innovative technology of anticancer therapy. However, organic-photosensitizers-based PTT/PDT exhibit some limitations for inducing effective immune responses, such as limited penetration depth of NIR [66], limited ICD effects [67], and limited concentration of photosensitizers in target tissues [68]. Compared with organic photosensitizers, various advantages are shown by inorganic nanomaterial photosensitizers, such as gold nanomaterials, graphene oxide, Prussian blue nanoparticles, and BP. For example, the reported advantages of inorganic nanomaterials include low cost, targetability, enhanced permeability, improved permeability and retention (EPR) effects (<200 nm) and recruitment of immunocytes, photodegradation, sensitive NIR reactivity, and a significant extinction coefficient [69–71]. In recent years, nanomaterials with inherent physicochemical properties, such as thermal conductivity and optical properties, were reported to mediate PTT/PDT [72].

BP, characterized by a band gap, in-plane anisotropy, biocompatibility, and biodegradability, has been widely reported to produce heat and ^1^O_2_ as one of the components of ROS under NIR laser [27]. For example, in 2016, Shao et al. concluded that PEG-modified BPQDs reveal potential clinical effects. When tumor-bearing mice treated PEG-modified BPQDs with NIR, they discovered that the temperature in tumor site was increased by 26.3°C within 10 minutes, even reaching a maximum temperature of 54.4°C, which is enough to ablate tumor cells [73]. Guo and colleagues firstly reported that BPQDs produce efficient ROS under NIR irradiation to achieve anticancer potential [74]. With intense research, more and more strategies are being used to improve heat and ROS conversion efficiency of BP-based PTT/PDT. BP functions are the most commonly strategies, including polymers functionalization [75], metal functionalization [76, 77], and nanoparticles coating [78]. For example, Jia et al. used Au-thiosugar to functionalize BP in a new study, and they found that metal ion modified BP exhibits a narrower band gap, which enhances thermal conversion efficiency [79].

### 4.2. BP-Based Sonodynamic Therapy

As mentioned above, although BP as inorganic photosensitizers can enhance sensitive NIR reactivity, the penetration of NIR is always limited. Recently, multiple research groups have confirmed that piezoelectric BP under ultrasound irradiation can be used as sonosensitive agents to generate ROS to damage cancer cells, defined as sonodynamic therapy (SDT) [80, 81]. Compared with NIR irradiation, ultrasound irradiation shows deeper tissue penetration, which provides potential to enhance the conversion efficiency of ultrasound for amplified ROS generation. With BP-based SDT as a novel antitumor modality, more and more strategies are being explored to enhance the generation efficiency of ROS. Liu et al. discovered that covalent modification, especially benzoic-acid-functionalized BP, can promote the formation of OH^−^ as one of the components of ROS [82]. On the side, Chen's team employed Au-anchored BP to enhance sensitivity of sound sonosensitizers and employed MnO_2_ shell encapsulated BP to enhance antioxidant depletion, both of which amplified the generation efficiency of ROS [83]. Therefore, SDT is another major innovation followed phototherapy and gives new opportunities for clinical antitumor therapy. And in situ vaccine induced by SDT may also have stronger immunogenicity, which also brings a hot area of BP-based immunotherapy.

### 4.3. BP-Based Photoacoustic Therapy

BP as photoacoustic-imaging contrast agent was demonstrated to achieve efficient and safe tumor diagnosis [25]. BP under NIR irradiation can transform light energy into heat causing nano-hole near the nanoparticles to expand and collapse, which produces ultrasonic radiation. The successful development of BP-based photoacoustic imaging not only provides a novel technology for cancer photoacoustic imaging diagnosis, but also gives prospective regimen for cancer precise treatment. Well actually, the photoacoustic shockwaves were activated by nanoparticle under NIR irradiation effective therapeutic effect for cancer precise elimination, which is called photoacoustic therapy (PAT) [84]. Different from PDT with limited ROS yield and PTT with overheat, BP-based PAT shockwave generation can achieve precise attack on the tumor site. In Zeng's study, they prepared multifunctional BP nanoparticles targeting mitochondria, and shockwave generated by the nanoparticles under the action of PAT produced the precise destruction to mitochondria and induced effective ICD effects [85]. Therefore, it can be concluded that PAT may bring a new round of innovation in precision cancer treatment.

### 4.4. BP-Based Photoimmunotherapy

Known for its natural antitumor biological activity, BP can be endocytosed into tumor cells, which are characterized by intense intracellular oxidative stress and accelerated energy metabolism, to degrade rapidly into phosphate anions and induce apoptosis of cancer cells [86]. BP has also shown therapeutic effects against cancer in biological imaging, drug delivery, and phototherapy, as shown in Figure 5(a). What is more, BP-based phototherapy, including PTT, PDT, PAT, and SDT, can cause a “double-kill” to tumor cells by converting NIR into heat, ROS, or shockwave to directly damage cancer cells and subsequently inducing an antitumor immune response, which is defined as PIT [87, 88]. As shown in Figure 4(b), BP-based phototherapy leads to the release of tumor-associated antigens (TAAs), which stimulate the maturation of dendritic cells (DCs) to induce an antigen-specific cytotoxic T cells (CTLs) response, called PIT. As with other photosensitizers, BP-based PIT causes ICD, facilitating the construction of an in situ vaccine in local tumors [89]. First, the TAAs released from damaged tumor cells are presented to naive T cells by DCs to induce a CTLs response, which overcomes the low immunogenicity of most cancer vaccines and heterogeneity of mutated neoantigens [66, 90]. Second, PIT-induced ICD promotes the release of damage-associated molecular patterns (DAMPs) [91, 92], such as calreticulin (CRT), adenosine triphosphate (ATP), high-mobility group box 1 (HMGB1), and heat shock proteins (HSPs), which is essential for maturation and infiltration of DCs. To be more specific, CRT facilitates the phagocytosis of macrophages and DCs, HMGB1 and HSPs facilitate maturation of DCs, and ATP facilitates the infiltration of DCs into tumor sites [66, 93]. Third, PTT also can reverse the immunosuppression of the TME by promoting immune cells, such as DCs, T cells, B cells, and natural killer cells, to infiltrate into the TME [66, 94–96].

## 5. The Potential of BP in Immunotherapy

### 5.1. BP-Based Nanovaccine

Tumor vaccines in multiple forms of tumor antigens, such as tumor lysates, TAAs, proteins, peptides, cellular vaccines, and nucleic acids, are mainly employed to induce an antigen-specific CTLs immune response against cancer [97]. Although a large number of cancer vaccines have been put into clinical trials, they failed in phase 3 due to lack of clinical efficacy [98]. Many obstacles, such as limited recognition of neoantigens, tumor immune tolerance, and significant individual variation of neoantigens in patients, can affect the immune response outcome of vaccines [99]. Therefore, the development of mutated neoantigens, the application of nanotechnology, and a combination of therapies will be important directions for the development of personalized cancer vaccines in the future. Recently, tumor cell membranes or exosomes, which accurately mimic the surface of tumor cells and completely retain numerous known and unknown TAAs of cancer calls, were employed to coat nanoparticles and construct nanovaccines, providing an opportunity for the research of personalized vaccines. In 2014, Fang et al. reported that nanovaccines constructed by cancer cell membrane-coated PLGA nanoparticles provided two antitumor modes delivering antigens to DCs and targeting tumor cells [100].

As a promising photosensitive nanomaterial, BP has shown great potential in the construction of nanovaccines in recent years. Scientists have constructed hyaluronic acid (HA) hydrogel-sustained delivery systems to encapsulate adjuvant and BP-based nanovaccines, which were prepared by coating BPQDs with a membrane of 4T1-luc cells, B16F10-luc cells, or surgical tumor cells [101]. The researchers found that the hydrogel-encapsulated nanovaccine systems irradiated with NIR promoted the recruitment and maturation of DCs at the tumor site. When combined with anti-PD-1 antibodies, the systems irradiated with NIR inhibited the recurrence and metastasis of a 4T1-luc breast tumor model and B16F10-luc melanoma tumor model. Zhao and colleagues utilized BPQDs coated by homologous targeting of cancer cell membranes to construct a similar nanovaccine [102]. When combined with anti-PD-L1 antibodies, the nanovaccines also showed the desired tumor immune response in vitro and in vivo [102]. Exosomes, as natural nanoparticles secreted from tumor cells, exhibit a variety of advantages when used as delivery systems, including homologous targeting ability, nontoxicity, excellent biocompatibility, high drug carrying capacity, and low or no immunogenicity [103]. In 2020, researchers from China prepared photo-nanovaccines by employing exosomes from the serum of tumor-bearing mice treated with hyperthermia of BPQDs [104]. This exosome not only did not affect the photothermal effect of BPQDs, but also prolonged the action time of BPQDs. The exosome-coated BPQDs with NIR not only showed prophylactic effect, but also revealed therapeutic effect to enhance the infiltration of lymphocytes, such as CD4^+^ and CD8^+^T cells, into the tumor site and the secretion of IFN-*γ* and TNF-*α* in LLC-bearing mice.

### 5.2. BP-Based Nanoadjuvant

As essential elements of tumor vaccines, adjuvants can make up for the low immunogenicity of tumor antigens and enhance the immune response through a variety of mechanisms, including promoting uptake cross-presentation and maturation of DCs, enhancing T cell proliferation, and regulating the immunosuppression of the TME [105]. Adjuvants are often divided into three categories [106]: (i) delivery systems (liposomes, virosomes, emulsions, polymeric particles, etc.), (ii) immunostimulants (TLR ligands, ISCOMs, etc.), and (iii) combination adjuvants (TLR9 + STING ligands, adjuvant systems, etc.). Nanoparticles with biosafety properties can not only serve as targeted delivery carriers for tumor antigens to protect them from degradation in the physiological environment, but also mimic the granular form of microbes to stimulate the immune system [107]. As 2D nanomaterials with excellent optical properties, they have also shown excellent potential as an adjuvant in recent years. For example, Yan et al. reported that chitosan-decorated graphene as an adjuvant promoted the release of cytokines and the activation of macrophages [108]. With good biosafety, BP nanosheets as adjuvants were reported to improve the effect of antitumor immunotherapy [109]. In the absence of any immune stimulants, the team employed CD8^+^T cell epitope peptides as vaccines to modify BP nanosheets. Their results confirmed that BPs play the role of adjuvant to promote DCs processing for antigenic peptides, including uptake, cross-presentation, and maturation of DCs by activation of the NF-*κ*Bp65 pathway. Notably, they discovered that BP not only promoted peptide-specific CD8^+^T cell invasion in spleen and tumor tissue, but also induced a Th1-type immune response.

### 5.3. BP-Based PIT Driven Necroptosis

Traditionally, cell death was divided into two categories, apoptosis and necrosis. Apoptosis, also called programmed cell death, is a physiologically active death of cells characterized by cell shrinkage, chromatin concentration, formation of apoptotic bodies, phagocytosis, and noninflammatory properties. In contrast to apoptosis, necrosis is an unregulated passive death of cells due to infection or injury with cellular swelling, release of cell debris, and inflammation [110]. However, there is increasing evidence that at least one type of necrosis, termed necroptosis, is programmed. Necroptosis is controlled by the interaction between protein kinase 1/3 (RIPK1/3) and mixed lineage kinase domain-like (MLKL) [111]. With the tolerance of cancer to apoptosis, necroptosis, which is characterized by immunogenicity and inflammation, has gradually received researchers' attention in antitumor immunotherapy [112]. However, necroptosis is a double-edged sword since it can also promote tumor proliferation and metastasis [113, 114]. While researching necroptosis for antitumor therapy, experts discovered that it can be induced by anticancer agents (etoposide, taxol, staurosporine, etc.) and proapoptotic agents (TRAIL, apoptosis proteins inhibitors, etc.) [113]. In fact, apoptotic ICD induced by BP-based PIT has been widely reported [115]. Zhao et al. precisely regulated certain parameters, such as irradiated time, spectrum, and concentration of BP, to generate a BP-based thermal therapy to induce necroptotic ICD [116]. They found that BP-based thermal therapy can induce necroptotic ICD when the BP concentration was 60 *μ*g/mL, and the irradiated time was 180 s. Western blotting assay verified RIP1 and RIP3 were highly expressed in model cells treated by BP nanosheets with optimal parameters. In response to necroptosis, the expression of Caspase-8, which can trigger apoptosis [117], did not change significantly. It was also further confirmed in their research that necroptotic ICD exhibited immunogenicity accompanied with the release of DAMPs, especially CRT, HMGB1, and ATP. Necroptotic ICD induced by BP nanosheets with optimal parameters led to a significant antitumor immune response, particularly in combination with adjuvants.

### 5.4. BP-Based PIT Combined with T Cell Immunotherapy

T cell immunotherapy, focused on immune checkpoint agents, gives hope to cancer patients. T cell immune checkpoint agents are mainly divided into inhibitors, which are represented by anti-CTLA-4 or anti-PD-1/PD-L1 and activators, which are still in the clinical research stage [118, 119]. However, the efficacy of T cell immune checkpoint blockades as monotherapy is only about 30% [120]. During the development and metastasis of tumors, tumor cells in complex TMEs escape the attack of CTLs by upregulating the expression of PD-L1, which binds with PD-1 to induce dysfunction and apoptosis of CTLs [121]. Therefore, synergistic combinations of nanomedicine with immune checkpoint agents may offer an opportunity to reverse TME immunosuppression and enhance T cell immunotherapy. For example, Nguyen et al. successfully employed BP to deliver PD-L1 inhibitor peptides into HCT-116 and B-16 cells, which significantly inhibited the expression of PD-L1 on tumor cells [122]. Researchers from different teams demonstrated that when combined with anti-PD-L1 antibodies, PIT benefitting from BPQDs effectively inhibited the growth and metastasis of triple-negative breast cancers by increasing the synergistic immunotherapy effect [48, 102]. Compared with PD-1/PD-L1 blockades, CTLA4 inhibitors can significantly inhibit regulatory T cells (Tregs), which promote the immune escape of tumor cells. BP-based PIT combined with CTLA4 inhibitors could significantly inhibit Tregs-mediated immunosuppression with an increase of the ratios of CD8+ CTLs/Tregs and CD4+ Teff/Tregs. Moreover, combination therapy also elicited a memory CTL immune response that prevented recurrence and metastasis of tumors [85].

### 5.5. BP-Based PIT Combined with Macrophage Immunotherapy

It is widely known that tumor-associated macrophages (TAMs) not only prevent T cells from attacking tumor cells, but also promote invasion, proliferation, and metastasis of tumor cells and facilitate the formation of angiogenesis in TME [123]. However, studies have confirmed that TAMs also can play another role that has antitumor effects [124]. TAMs can be divided into M1 TAMs and M2 TAMs based on phenotype and function, as shown in Figure 6. M1 TAMs secrete immunostimulatory and proinflammatory cytokines and chemokines, including TNF-*α*, L-6, IL-12, IL-23, CXCL9, and CXCL10 [123, 125–127]. M1 TAMs play antitumor roles in two main ways: (i) releasing toxicants such as nitric oxide (NO) and ROS to directly kill tumor cells, and (ii) exerting an immunostimulatory effect such as inhibiting Tregs and promoting antibody-dependent cell-mediated cytotoxicity (ADCC) and complement dependent toxicity (CDC), as well as antigen presentation [127, 128]. In contrast to M1 TAMs, M2 TAMs secrete immunosuppressive and anti-inflammatory cytokines and chemokines, including IL-4, IL-10, IL-13, CCL22, and CCL24, and promote the invasion, proliferation, and metastasis of tumor cells [123, 125, 127]. Compared to the low infiltration of T cells, it is noteworthy that TAMs constitute the majority of the infiltrating immune cells in the TME [126]. Researchers have, therefore, recognized that TAMs can be used as a target of antitumor immunotherapy. Currently, macrophage-based immunotherapy can be roughly divided into five types: (i) inhibition of recruitment at tumor site, (ii) reprogramming of polarized macrophages from M2 to M1, (iii) reduction of M2 TAMs in TMEs, (iv) application of nanoparticles, and (v) repairing of antitumor activity of macrophages [129].

Although M1 TAMs possess the ability to kill tumor cells, the clever tumor cells can express CD47, which binds to SIRP*α* on the macrophage surface to release the signal: “do not eat me” [130]. Therefore, immunotherapy that blocks the CD47/SIRP*α* pathway to repair antitumor activity of M1 TAM has become a new research strategy. Figure 6 shows the repair of antitumor activity involves mechanisms including the following: (i) eliminating the “do not eat me” signal, (ii) promoting tumor antigen presentation by DCs, (iii) mediating ADCC and CDC, and (iv) inducing apoptosis of tumor cells [131]. However, while a large number of inhibitors targeting immune checkpoint CD47-SIRP*α*, especially anti-CD47 antibodies, have been tested in preclinical and clinical trials, the antitumor activity of single agents is not always obvious and accompanied by side effects such as the reduction of red blood cells [132]. The combination of CD47/SIRPA-blocking agents with other antitumor immunotherapies is a promising development to enhance the antitumor activity of macrophage immunotherapy. Xie et al. discovered that BP-based photothermal treatment can promote the activity of anti-CD47 antibody-induced macrophage immunotherapy [133]. In addition to directly blocking the “do not eat me” CD47/SIRP*α* pathway, the BP-based photothermal treatment combined with anti-CD47 antibodies also enhances the polarization of TAMs into M1 TAMs in primary and metastasis tumor sites to induce antitumor activity. As mentioned above, M1 TAMs enhance the presentation of TAMs to further promote CTLs responses with an increase in the secretion of cytokines such as IL-6, IFN-*γ*, CCL2, and CXCL9. In short, BP-based photothermal treatment combined with anti-CD47 antibodies produces a synergistic antitumor immune response.

In addition to promoting macrophage immunotherapy when used in combination with CD47/SIRPA blockers, BP nanoparticles can also be used to deliver drugs such as siRNA to increase M1 TAMs or inhibit M2 TAMs at tumor sites. For example, HA-modified BP has the ability to polarize macrophages from M2 TAMs to M1 TAMs with an increased release of IL-2 [115]. Mo's team explored the mechanism of macrophage polarization and discovered that BP nanosheets coated with corona binding to STIM2 promoted Ca^2+^ influx, which activated p38 MAPK and NF-*κ*B p65 [134]. The polarized M1 macrophages benefitting from corona-coated BP promoted the killing ability of macrophages through direct or indirect ways. In another study, nanosystems of BP-delivered interleukin-1*α*-silencing siRNA inhibit regulatory T cell (Treg) infiltration into TMEs by enhancing the secretion of CCL-22 [135]. Although silver ions (Ag^+^) exhibit inhibitory activity on pathogenic bacteria and tumor cells, the physiological stability and targeting ability of Ag^+^ are poor. As a result, researchers found that Ag-coupled BPQDs promote the release of Ag^+^ under NIR laser irradiation and enhance the phagocytosis of Ag^+^ by macrophages at tumor sites, which further motivates the release of inflammatory factors such as TNF-*α* and IL-6 to enhance the immunogenicity of ICD [28]. And the BP-based immunotherapeutic potentials described above are summarized in Table 2.

## 6. Advantages of BP Compared with Graphene in Nanomedicine

Compared with BP, graphene as 2D material is composed of carbon atoms with an sp^2^-hybridized monatomic layer structure. Graphene, and especially its derivatives, exhibits great prospects in nanoelectronic applications, catalysts, nanomedicine, environmental areas, and other fields [136–138]. However, since structure determines properties, graphene possesses two obvious disadvantages involving zero band gap and cytotoxicity when compared with BP [20, 135]. Bilayer-structural monolayer BP possesses a direct-gap (0.3–2 eV) semiconductor that converts electronic signals into light. More importantly, the band gap of BP can be adjusted to promote a wide range of light absorption ranging from visible to mid-IR [23, 139]. Therefore, the band gap of BP lays a firm foundation for its application in nanomedicine, such as for photothermal therapy and photodynamic therapy. Although graphene has shown promising therapeutic effects in tumor therapy, including immunotherapy and photothermal therapy, researchers have noted that graphene generates undesirable cytotoxicity based on carbon in application. Syama et al. reported that graphene derivatives, such as GO and reduced GO, could cause cell membrane damage and cytotoxicity based on oxidative stress, as well as DNA damage [140]. Fortunately, it was found that BP composed of phosphorus atoms can be converted into a phosphate form under physiological conditions, which promotes the biocompatibility, biodegradability, and low-toxicity of BP in nanomedical applications [34].

## 7. Limitations of BP in Nanomedicine

Although 2D BP materials with unique structures, properties, and functions show great application prospects in the field of nanomedicine, some limitations of this material have been discovered. First, as the preparation of BP is still in the preliminary stage of exploration, industrialization remains extremely challenging. Second, BP exposed to air promptly reacts with oxygen and water. Therefore, improving its stability has become the key issue to promote the practical application of BP. Developing new passivation methods to improve the long-term stability of BP could be an effective measure. Third, since the mechanism of cytotoxicity induced by BP is extremely complex, it is important to evaluate the safety of BP for biomedical applications. Although BP can damage cell membranes and intracellular organelles through its unique photothermal or photodynamic properties, its ability to target tissues depends on many factors, such as materials concentration, nano-size, and morphology. Fourth, BP is a double-edged sword, as it can both promote and inhibit antitumor immune responses, such as its protumor and antitumor effects on macrophages. For these reasons, precise design of the structure and function of BP is essential to promote its application in nanomedicine.

## 8. Conclusion

Although graphene-based hyperthermia has given new hope to cancer patients, two notable disadvantages of graphene are its zero-band gap and cytotoxicity. Recently, supermaterial BP has shown great potential in the fields of optoelectronics and biology when benefitted by a puckered bilayer structure of phosphorus atoms. Contrary to the cytotoxicity of graphene, BP is biodegradable and biocompatible, which lays the foundation for its application in cancer treatment. As mentioned above, BP not only possesses natural anticancer biological activity, but also exhibits PTT/PDT effect with NIR. Specifically, the increased ROS generation and shockwaves initiated by BP-based SDT/PAT under ultrasound or NIR irradiation enhance the killing of tumor cells. This is followed by the release of TAAs from the killed tumor cells, which activates an antitumor immune response to cause a “double-kill” to tumor cells. BP has, therefore, been widely studied as a nanovaccine, nanoadjuvant, and combined immunotherapy regimen in recent years. In short, BP creates a novel technology for nano-diagnosis and nano-treatment, which has the advantages of real-time monitoring and precision treatment of diverse and dynamic as well as heterogeneous cancers.

## Figures and Tables

**Figure 1:** The potential application of BP in immunotherapy.

**Figure 2:** The structure of BP. Abbreviations: (a) the 3D structure of BP; (b) the lateral view of BP; (c) the top view of BP; *x* armchair; *y* zigzag.

**Figure 3:** The degradation mechanism of BP.

**Figure 4:** The passivation techniques of BP.

**Figure 5:** The application of BP in biomedicine. (a)BP exhibit natural antitumor biological activity, biological imaging, drug delivery, and phototherapy (including PAT, PDT, and PTT). (b) PIT is induced by BP. Shockwaves, ROS, or heat activated by BP with INR irradiation cause structural damage of tumor cells. These damaged tumor cells release TAA, which facilitates the construction of in situ vaccines. This in situ vaccine promotes the maturation of DC, which induced the generation, proliferation, and infiltration of cytotoxic T cells benefit by DAMPs (including CRT, ATP, HMGB1, and HSPs). Abbreviations: BP, black phosphorus; PTT, photothermal therapy; PDT, photodynamic therapy; SDT, sonodynamic therapy; PAT, photoacoustic therapy; PIT, photoimmunotherapy; ROS, reactive oxygen species; NIR, near-infrared; TAAs, tumor-associated antigens; DCs, dendritic cells; CTLs, antigen-specific cytotoxic T cells; DAMPs, damage-associated molecular patterns; CRT, calreticulin; ATP, adenosine triphosphate; HMGB1, high-mobility group box 1; HSPs, heat shock proteins.

**Figure 6:** The effect of TAMs in tumor treatment. TAMs are divided into M1 TAMs and M2 TAMs. The M2 TAMs are protumor through secreting anti-inflammatory cytokines and chemokines, enhancing infiltration of Tregs in tumor site and inhibiting antigen presentation of DCs. The M1 TAMs are antitumor through enhancing polarization of M2 TAMs to M1 TAMs, secreting proinflammatory cytokines and chemokines as well as toxicant and blocking the CD47/SIRP*α* pathway. Abbreviations: TAMs, tumor-associated macrophages.

**Table 1:** The strategies of modifications on BP.

Functionalization	Interactions	Materials
Surface encapsulation	Coating	Polymers: PMMA, PHMA-co-ps, PIL-TFSI, PEG. Nanoparticle: WPU nanoparticles, hyaluronic acid hydrogel. Biomembrane: Red blood cell membranes, cancer cell membrane, platelet membrane 2D heterostructures: hBN, graphene, MoS2. Others: AlOx, SiO2.

Chemical modification	Nucleophilic substitution radical reaction nitrene addition	Covalent modification: Aryl diazonium, PDDF, Nile blue dye, aryl iodonium salts, azide, TiL4. Noncovalent modification: TCNQ, PDI, Ag+, PILs.

Element doping	Van der Waals interactions cation-*π* interactions electrostatic interactions	TCNQ, PDI, anthraquinone, Ag^+^, PILs.

**Table 2:** The potential of BP in immunotherapy.

Nano-shape	Functionalization	Vaccine	Adjuvant	Size	Zeta potentials	Combination therapies	Outcomes	Reference
BPQDs	Encapsulation of BP with tumor cell membrane	Tumor cell membrane encapsulated BPQDs	LPS (lipopolysaccharide)	120 nm	−23 mV	PD-1 checkpoint blockade antibody	1. Stimulating the expansion and maturation of DCs; 2. Enhancing tumor-specific CTLs to eliminate the residual and metastatic tumor when combined with PD-1 antibody.	[101]

BPQDs	Encapsulation of BP with tumor cell membrane	Tumor cell membrane encapsulated BPQDs		30 nm	−24.1 mV	PD-1 checkpoint blockade antibody	1. Inducing maturation of DCs; 2. Promoting the local and systemic antitumor immune response.	[102]

BPQDs	Encapsulation of BP with exosomes	Exosomes encapsulated BPQDs		100 nm			1. Promoting differentiation and maturation and infiltration of T lymphocytes into the tumor tissue.	[104]

BP nanosheets	Noncovalent modifications of BP with phenylalanine-lysine-phenylalanine (FKF) tripeptide-modified antigen epitopes	Antigen peptide (OVAp)	BP	34 nm			1. Enhancing drug delivery, DCs activation and Th1-type immune response.	[109]

BP nanosheets	Modifications of BP with bPEI-PEG	TAAs released from tumor cells treated with BP (in situ vaccine)	CpG				1. Driving necroptosis in ablated tumor cells to exhibit considerable immunogenicity.	[116]

BP nanosheets	Encapsulation of BP with cholesterol-polyethylene glycol-poly-l-lysine	In situ vaccine		235.9 nm	−21.9 mV	PD-1 inhibitor peptide	1. Exhibiting targeted and promised cancer immunotherapy by combination therapies.	[122]

BPQDs	Encapsulation of BP with erythrocyte membrane	In situ vaccine		100 nm	−17 mV∼−13 mV	PD-1 checkpoint blockade antibody	1. Delaying residual and metastatic tumor growth by combination therapies; 2. Increasing the infiltration and activity of CD8+ T cells in the tumor by combination therapies.	[48]

BP nanosheets	Modifications of BP with HS-PEG-NH2	In situ vaccine	Toll-like receptor 7 and 8 (TLR7/TLR8) agonist (resiquimod R848)	65 nm		anti-CTLA-4 antibody	1. Promoting the infiltrating CD8+and CD4+ T-cells; 2. Inhibiting the growth of distant tumors; 3. Increasing the number of memory T cells.	[85]

BP nanosheets	Modifications of BP with PEG-NH2	In situ vaccine		100∼200 nm		anti-CD47 antibody	1. Inducing repolarization of TAMs to M1 TAMs; 2. Promoting cross-presentation of TAAs to activate CTLs activity.	[133]

BP nanosheets	Encapsulation of BP with plasma proteins	In situ vaccine		207 nm	−4.85 mV		1. Facilitating M1 TAMs formation by BP nanosheets coated with corona binding to STIM2 to promote Ca2+ influx; 2. Promoting cellular cytotoxicity and effective phagocytosis of cancer cells.	[134]

BP nanosheets	Modifications of BP with poly-L-histidine	In situ vaccine		<200 nm			1. Inhibiting the secretion of CCL-22 which represent M2 TAMs chemokines by BP-delivered interleukin-1*α* silencing siRNA.	[135]

BPQDs	Modifications of BP with three polymers, including PEG, polyacrylic acid (PAA) with an Ag + ions-trapping function, reactive oxygen species (ROS)-sensitive polypropylene sulfide (PPS)	In situ vaccine		<200 nm			1. Motivating release of inflammatory factors such as TNF-*α* and IL-6 to enhance the immunogenicity of ICD by enhancing phagocytosis of Ag^+^ released from BP at tumor site.	[28]

## Data Availability

No new data were created or analyzed in this study. Data sharing is not applicable to this article.

## Abbreviation

BP: Black phosphorus
NIR: Near-infrared
ROS: Reactive oxygen species
PTT: Photothermal therapy
PDT: Photodynamic therapy
SDT: Sonodynamic therapy
PAT: Photoacoustic therapy
PIT: Photoimmunotherapy
TME: Tumor microenvironment
rGO-Au: Reduced graphene oxide modified with Au
ICD: Immunogenic cell death
2D: Two-dimensional
BPQDs: BP quantum dots
PMMA: Polymethyl methacrylate
PHMA-co-PS: Poly (2-hydroxyethyl methacrylate)-co-poly (styrene)
PIL-TFSI: Poly (1-hexyl-3-vinylimidazolium) hexafluorophosphate salt
PEG: Poly (ethylene glycol)
WPU: Polyurethane
hBN: Hexagonal boron nitride
4-NBD: 4-Nitrobenzenediazonium salts
4-MBD: 4-Methoxybenzenediazonium tetrafluoroborate salts
PDDF: Poly[(1,4-diethynylbenzene)-alt-9,9-bis (4-diphenylaminophenyl) fluorene]
TiL4@BPs: Titanium sulfonate ligand (TiL4) coordinated BP
TCNQ: 7,7,8,8-tetracyano-p-quinodimethane
PDI: Perylene diimides
Ag+: Silver ions
CBM: Conduction band minimum
EPR: Permeability and retention
TAAs: Tumor-associated antigens
DCs: Dendritic cells
CTLs: Antigen-specific cytotoxic T cell
DAMPs: Damage-associated molecular patterns
CRT: Calreticulin
ATP: Adenosine triphosphate
HMGB1: High-mobility group box 1
HSPs: Heat shock proteins
HA: Hyaluronic acid
RIPK1/3: Protein kinase 1/3
MLKL: Mixed lineage kinase domain-like
Tregs: T cells
TAMs: Tumor-associated macrophages
NO: Nitric oxide
ADCC: Antibody-dependent cell-mediated cytotoxicity
CDC: Complement dependent toxicity
LPS: Lipopolysaccharide
OVAp: Antigen peptide
FKF: Phenylalanine-lysine-phenylalanine
PAA: Polyacrylic acid
PPS: Polypropylene sulfide.
